# The Efficacy of Ultrasound-Guided Superior Laryngeal Nerve Block as an Adjuvant to General Anesthesia during Suspension Laryngoscopy Vocal Cord Polypectomy

**DOI:** 10.1155/2022/1594829

**Published:** 2022-06-28

**Authors:** Yu Zhou, Bin Chen, Yiqiang Xiong, Xiangdi Yu

**Affiliations:** ^1^Department of Anesthesiology, Zunyi Medical University, Zunyi, Guizhou, China; ^2^Department of Anesthesiology, Guizhou Provincial People's Hospital, The Affiliated Hospital of Guizhou University, Guiyang, Guizhou, China

## Abstract

**Background:**

In the current study, we assessed the effect of the ultrasound-guided internal branch of the upper laryngeal nerve (USG-guided iSLN) block combined with general anesthesia on perioperative sore throat (POST), cough, hoarseness of voice, intraoperative hemodynamic changes, and the quality of early recovery for the patients undergoing suspension laryngoscopy vocal cord polypectomy (SLVCP).

**Methods:**

This was a randomized controlled trail. Eighty patients, aged from 18 to 70 years old, ASA I ∼ II, scheduled for polypectomy of the vocal cord by using a laryngoscope, were randomized into 2 groups (*n* = 40 each) using a random number table. Patients in group C received general anesthesia (GA), whereas those in group S received USG-guided iSLN block bilaterally (37.5 mg of 0.375% ropivacaine, 5 ml each side) combined with GA. The primary outcome was the quality of patients' recovery using the Quality of Recovery Questionnaire (QoR-9). The secondary outcomes were postoperative cough, sore throat, hoarseness of voice, and hemodynamic changes in both groups at corresponding time points. The adverse reactions such as postoperative chocking, or aspiration, and dyspnea was recorded as well.

**Results:**

The QoR-9 scores of patients in group C were lower than those of group S at time points of D1∼D2 (*P* < 0.05). Patients in group S had a significantly lower incidence of perioperative cough than those in group C in the early postoperative period (1 hour after extubation) (*P* < 0.05), the scores of sore throat were lower in group S than those in group C (*P* < 0.05), the incidence of postoperative hoarseness was increased in group S than that in group C at the time points of 30 min, 2 h, and 4 h after extubation (*P* < 0.05); however, the incidence of postoperative hoarseness was decreased in group S than that in group C at the time point of 24 h after extubation (*P* < 0.05). MAP and HR of group S was lower than those of group C at time points of T1∼T4 (*P* < 0.05). No serious adverse events were observed in both groups.

**Conclusion:**

The study found that the application of ultrasound guided superior laryngeal nerve block combined with general anesthesia for the patients undergoing SLVCP could effectively promote the quality of early recovery. Clinical trial registration: This trial is registered with NCT05309174. The date of registration: March 12th 2021.Trial registry name: The Study of Bilateral Upper Laryngeal Nerve Block for Supporting the Removal of Vocal Cord Polyps Under Laryngoscopy.

## 1. Introduction

Vocal cord polyps are benign proliferative lesions, which are usually located unilaterally at the free edge of the vocal cord membrane [1]. The main cause of polyp formation is excessive vocalization and mechanical damage resulting from misuse or intense cough [2]. Chronic/recurrent upper respiratory tract infections, smoking, allergies, and extraesophageal reflux are cofactors. The presence of these lesions causes speech inefficiency and a range of phonological symptoms that can significantly affect the quality of life. Patients complained of hoarseness, voice fatigue, double tone, and inability to project sounds [3]. Suspension laryngoscopy vocal cord polypectomy (SLVCP) is commonly used to diagnose or treat benign or malignant diseases of the vocal cords [4]. To avoid the movement of cords, coughing, or bucking, the procedure is performed under general anesthesia, in which the adequate muscle relaxation and immobile vocal cords could meet the surgical requirement [5]. The challenge is the relatively short operating time that demands patient quick awaking and recovery of muscle power [2]. However, the paradox is that the larynx is a highly reflexogenic region, the stimulation of the pharynx gives rise to sympathetic excitation and the consequence is that the events such as tachycardia, hypertension, and arrhythmias may happen; which means that deep anesthesia is required to suppress stress response [6]. So, exploring a new technique that could inhibit the stress response and promote quick awaking is meaningful for the patients undergoing SLVCP.

The internal branch of the superior laryngeal nerve (iSLN) is paralleled by the superior laryngeal artery, which goes through the thyrohyoid membrane and dominates sensory sensation above the vocal cord [7]. Bilateral superior laryngeal nerve blocks provide anesthesia to the larynx above the vocal cords (the epiglottis, aryepiglottic folds, and laryngeal structures to the false cords). For this nerve block, the local anesthetics are infiltrated to the thyrohyoid membrane between the thyroid and hyoid cartilage [8]. This method of local nerve block is now widely used for fiberoptic bronchoscopy, laryngoscopy, and conscious intubation of difficult airway to reduce the hemodynamic change caused by airway stimulation and provide better practical conditions for operation [9–12]. Studies have shown that bilateral iSLN blocks can reduce cardiovascular response caused by the sympathetic stimulation during surgery [13] and reduce the incidence and severity of postoperative cough, sore throat, and hoarseness of voice [14, 15]. Therefore, it could be an ideal adjuvant to general anesthesia for SLVCP.

Our present study is a randomized controlled trial that is designed to investigate the effectiveness of ultrasound-guided iSLN (USG-guided iSLN) block as an adjuvant to general anesthesia for SLVCP. It was hypothesized that general anesthesia combined USG-guided iSLN block could improve quality of recovery for the patients undergoing SLVCP.

## 2. Materials and Methods

The study protocol was approved by the Ethics Committee of Guizhou Provincial People's Hospital and was performed according to the Declaration of Helsinki (1996) and all relevant Chinese laws. The trial was registered at https://register.clinicaltrials.gov (NCT05309174). Written informed content was obtained from all patients before inclusion.

### 2.1. Study Population and Randomization

This randomized controlled trial was approved by the Ethics Committee of Guizhou Provincial People's Hospital. Patients with local pathology of the neck, bleeding diathesis, allergy to local anesthetic agents, intellectual impairment, or psychiatric conditions including adequate communication and the body mass index≥30 kg/m2 were excluded from the study. A total of 80 patients, aged 18–65 years old, ASA physical status I or II, scheduled to undergo SLVCP, were randomly allocated to an USG-guided iSLN group (S group) or a control group (C group) at a 1 : 1 ratio using a random number table (Figure 1). Patients in group C received general anesthesia (GA), whereas those in group S received GA combined with USG-guided iSLN block bilaterally with 5 ml of 0.375% ropivacaine on either side.

### 2.2. Anesthesia Process

All participants presented to the operation room on the day of surgery after overnight fasting of 8 hours. When entering the operating room, participants are routinely monitored for heart rate (HR), oxygen saturation (SpO_2_), noninvasive blood pressure (NIBP), mean arterial pressure (MAP), electrocardiogram (ECG), heart rate (HR), and end-expiratory carbon dioxide partial pressure (PETCO_2_). At the same time, the patients were given 8 ml/kg·h lactated Ringer's solution intravenously. GA was induced with sufentanil (0.35 ug/kg), propofol (2 mg/kg), and cisatracurium (0.2 mg/kg). After a routine intravenous anesthetic induction, orotracheal intubation was performed. In general, the No.6.0 endotracheal tube was used for women and the No. 6.5 tube for men. USG-guided bilateral iSLN block with 0.375% ropivacaine, 5.0 ml on either side was given to all the patients in group S. Anesthesia was maintained using inhalation of sevoflurane (1.5%–3%), intravenous injection of propofol (5–7 mg·kg^−1^·h^−1^) and remifentanil (0.08–0.15 ug·kg^−1^·min^−1^) to maintain the surgery carried out normally. At the end of the surgery, anesthesia maintenance drugs were ceased when the laryngoscopy was withdrawn. Subsequently, patients were sent to the postanesthesia care unit (PACU) waiting for recovery.

### 2.3. Technique of USG-Guided iSLN Block

Patients in group S underwent USG-guided iSLN Block. By strict aseptic manipulation, the specific operation is as follows: patients took the supine position, with the neck extended. A high-frequency (6–13 MHz) ultrasound probe (Sonosite, USA) was placed over the thyroid cartilage area with a lateral orientation. The thyroid cartilage was identified, showing a hyperechoic signal on sonography. Next, the probe was moved to one side, closer to the cephalad level slightly. The thyrohyoid membrane was a hyperechoic line graph, and the nerve structure around the superior laryngeal artery was the internal branch of the superior laryngeal nerve (Figure 2(a)). The block was performed using a 24-gauge 1-inch needle with a 10 ml syringe that was filled with 0.375% ropivacaine. Aspiration was performed to detect either air or blood; then, an in-plane method was used to inject 0.375% ropivacaine (5.0 ml each side) bilaterally (Figure 2(b)), with local compression and observation for 3 minutes. The same technique was repeated on the other side.

### 2.4. Measures

To assess the cough severity, rating it from 0 to 4 on a 4-grade scale (Table 1) just before extubation (bucking on the ETT) and after extubation at 10 min, 2 h, and 4 h, the incidence of postoperative sore throat (POST) and hoarseness of voice was measured according to a 4-grade scale (Table 1) at 30 min, 2 h, 4 h, and 24 h following extubation. Grades 2 and 3 were regarded as severe cough, sore throat, and hoarseness of voice. The incidence of postoperative cough, sore throat, and hoarseness of voice was recorded according to the patients suffering from severe cough, sore throat, and hoarseness of voice (grades 2 and 3). The hemodynamic changes (MAP and HR) were also recorded at the following time points: before induction (T0), immediately after intubation (T1), immediately after the operation started to support laryngoscope exposure (T2), immediately after extubation (T3), and 5 min after extubation (T4). Meanwhile, patients' recovery scores were assessed using the 9-item quality of recovery score (QoR-9) [16, 17] on the operation day (D0) and the first day (D1) after operation. Moreover, operating time, awaking time of anesthesia, intraoperative opioid dosage, hospital stays, and complications such as dysphagia, dyspnea, and laryngospasm, were also recorded.

### 2.5. Statistical Analysis

According to sample size calculation in clinical research [18], the power (1 − *β*) was set at 0.8, the type I error rate was set at 5%, and the sample size was 40 for each group. The calculation was performed on the website http://powerandsamplesize.com. Continuous quantitative normally distributed data were expressed as the mean and standard deviation (SD). Qualitative nominal data, e.g., the incidence of complications was expressed as frequency or percentage. Quantitative discrete data were expressed as the median and range. Normally distributed data were analyzed using Students *t*-test and two-way ANOVA with repeated measures. The Mann–Whitney *U-*test was used for nonparametric data. Chi-square or Fisher's exact tests were used as appropriate to compare qualitative data. A *P* value <0.05 was considered statistically significant.

## 3. Result

### 3.1. General Data

This study included 80 patients who were scheduled to undergo suspension laryngoscopy vocal cord polypectomy with general anesthesia and the flowchart is presented in Figure 1. Demographic data, ASA status, and surgery times were comparable between the two groups of patients (Table 2). The duration of surgery showed no statistically significant difference between both groups as there was no difference between both groups regarding the postoperative silence time or the hospital stay (Table 2). However, anesthetic consumption such as sufentanil and remifentanil was less in group S than in group C (*P* < 0.05) (Table 2).

### 3.2. Primary Outcome

The QoR-9 scores of group S were 13.05 ± 1.80 on the operative day after operation and 16.75 ± 1.50 on the first day after operation; the QoR-9 scores of group C were 11.38 ± 2.47 on the operative day after operation and 15.10 ± 1.61 on the first day after operation. Compared with group C, the QoR-9 scores of group S were higher on *D*0 and *D*1(Table 3). Furthermore, the QoR-9 scores were increased from *D*0 to *D*1 in both groups (Table 3).

### 3.3. Secondary Outcome

Incidence of severe cough, incidence of severe postoperative sore throat (POST), and incidence and severity of postoperative hoarseness of voice at different time points between the two groups are the secondary outcome. The incidence and severity of perioperative cough in Group S were lower than those in Group C (*P* < 0.05) (Table 4). The analgesic effect of sore throat in Group S was significantly better than that in Group C in the postoperative period (*P* < 0.05) (Table 5). The hoarseness was better in group C as less frequent and lower severity hoarseness occurred than that in group S in the early postoperative period. However, 4 hour postextubation, the incidence, and severity of hoarseness in group S are significantly reduced (*P* < 0.05) (Table 6).

### 3.4. Hemodynamics at Different Time Points between the Two Groups

The hemodynamic responses of the two groups were comparable in terms of perioperative hemodynamic responses (*P* < 0.05) (Figures 3 and 4). The MAP and HR of group S remained significantly lower than those of Group C at *T*1, *T*2, *T*3, and *T*4 (*P* < 0.05) (Tables 7 and 8). At these time points, a maximum increase in blood pressure and the heart rate was observed at T1.

## 4. Discussion

Our present study demonstrated that the application of ultrasound-guided superior laryngeal nerve block combined with general anesthesia for the patients undergoing SLVCP could effectively promote the quality of early recovery. In addition, it could also maintain hemodynamic stability, reduce the usage of opioids, decrease the incidence and severity of cough, sore throat, and hoarseness and facilitate patients' quick awaking.

SLVCP is the category of minor surgery, and the patients wish to recover quicky to be back to their normal life. However, the most patients undergoing SLVCP are often disturbed by cough, sore throat, and hoarseness [4], and the complications after surgery are not conducive to the patients' recovery [19]. Although the occurrence of postoperative cough, sore throat, and hoarseness of voice can be reduced by choosing a smaller type of an endotracheal tube, using appropriate pressure of tracheal cuff, intravenous or topical lidocaine [20], lidocaine into the endotracheal tube cuff [21], and anti-inflammatory agents such as steroids [8, 22,23]. However, all the aforementioned measures are not satisfactory. In addition, the placement of suspension laryngoscopy is often accompanied by severe sympathetic stimulation, which is extremely hazardous for the patients with cardiovascular disease. Many techniques have been designed to find out possible approaches to reduce the occurrence of perioperative stress response, such as a topical local anesthetic (LA) to the laryngeal mucosa, administration of intravenous (IV) LA, short-acting opioids, or beta-adrenergic antagonists [24, 25]. However, the stress response could not be inhibited effectively by these approaches.

The iSLN is paralleled by the superior laryngeal artery, which passes through the thyrohyoid membrane and is divided into many small branches to the pharynx, the epiglottis, and the sensory nerve of the laryngeal mucosa above the glottic fissure [7]. The sensory innervation of the larynx is provided by the iSLN block which can be blocked bilaterally. Some studies have also shown that the iSLN block with lidocaine and steroids is an effective alternative to neuromodulators for patients with neurogenic cough [26]. And the application of the iSLN block is also becoming more and more extensive in support laryngoscopic surgery, as an adjuvant to general anesthesia, with the latter offering superior hemodynamic stability and less patient discomfort [27]. The present study is consistent with the previous ones, and the application of the bilateral iSLN block combined with general anesthesia could effectively offer superior hemodynamic stability during operation and promote the quality of early recovery postoperatively for the patients undergoing SLVCP. Usually, this block is performed blindly by recognizing the greater horn of the hyoid bone and the superior horn of the thyroid cartilage as anatomic landmarks [28]. With the clinical application and popularization of ultrasonography (US), US has already been applied to assist the performance of the iSLN block, which is capable of providing detailed imaging of the airway and adjacent anatomy [29]. The application of US guarantees the precise and effectiveness of the iSLN for each patient, and all patients tolerated the operation well without complications in our study.

In addition, we also found that the bilateral iSLN block could significantly reduce the incidence and severity of cough, decrease the sore throat score significantly within 24 hours postoperatively. Although the hoarseness was more serious in patients who received ultrasound-guided superior laryngeal nerve block in the early postoperative period, the degree of hoarseness was significantly relieved 24 hours after extubation. Consistent with our findings, the previous study demonstrated that the USG-guided iSLN block as an adjunct to GA significantly reduced postoperative cough, sore throat, and hoarseness [5].

### 4.1. Limitations

This trial has several limitations. First, we used single-concentration and single-dose local anesthetics in this study, and further study of the optimal concentration and dosage of local anesthetics is needed. Second, considering that resection of vocal polyp by using a suspension laryngoscope is generally relatively short, and the study did not monitor the depth of intraoperative anesthesia. It was judged and managed based on intraoperative blood pressure, heart rate, and clinical signs empirically, so the depth of intraoperative anesthesia may not meet the standard of unified quantification extremely well. Given the patient in good general condition, the study did not monitor invasive blood pressure, and intraoperative blood pressure may not be able to be reflected in a very timely and accurate manner. Future investigations could aim to find more efficient and accurate monitoring methods. Finally, the sample size is not large enough as well. A larger study would better elucidate the efficacy of the USG-guided iSLN block.

## 5. Conclusions

In this study, we provided evidence that the ultrasound-guided superior laryngeal nerve block could alleviate the incidence and severity of postoperative cough, sore throat, and hoarseness in patients compared with general anesthesia alone, providing a smoother hemodynamic response and a higher quality score for postoperative recovery.

## Figures and Tables

**Figure 1:** Patient recruitment, randomization, and follow-up in the trial.

**Figure 2:** The figure shows ultrasound images. The red line in (a) shows the area of the thyrohyoid membrane, and the red circle in (a) shows the area of the internal branch of the superior laryngeal nerve and the superior laryngeal artery. The arrow in (b) shows the puncture needle.

**Figure 3:** Mean arterial pressure (MAP) comparison of two groups at different time points. ^*∗*^=*P* < 0.05 vs. group C.

**Figure 4:** Heart rate (HR) of two groups at different time points. ^*∗*^=*P* < 0.05 vs. group C.

**Table 1:** Scoring system for severity of cough, sore throat, and hoarseness.

Score
*Cough severity*
Grade 0: no cough
Grade 1: light or single cough
Grade 2: more than one episode of unsustained (65 s) coughing
Grade 3: sustained (65 s) and repetitive cough with the left head

*Sore throat severity*
Grade 0: no sore throat
Grade 1: mild (complained of sore throat only upon inquiry)
Grade 2: moderate (complained of sore throat on his/her own)
Grade 3: severe (severe pain associated with a marked change in voice)

*Hoarseness severity*
Grade 0: none
Grade 1: noted by the patient
Grade 2: obvious to the observer
Grade 3: aphonia

**Table 2:** Characteristics and surgical details of the study population.

Characteristics	Group C	Group S	*p* value
Age (years)	45.73 ± 12.19	45.60 ± 12.16	0.964
Gender (M/F)	19/21	16/24	0.499
Height (cm)	163.73 ± 7.65	161.00 ± 8.75	0.142
Weight (kg)	63.43 ± 12.51	61.10 ± 10.95	0.379
ASA status (I/II)	0/40	0/40	
Hypertension (%)	3 (7.5)	3 (7.5)	1.000
Duration of surgery (min)	19.20 ± 11.42	18.98 ± 10.66	0.928
Postoperative silence time (min)	65.25 ± 70.97	59.70 ± 63.70	0.714
Hospital stay (days)	4.13 ± 1.44	4.08 ± 1.33	0.872

*Anesthetic*			
Sufentanil (ug)	23.63 ± 5.77	23.50 ± 6.91	0.930
Remifentanil (mg)	0.05 ± 0.09	0.04 ± 0.09	0.592

Data are expressed as the mean ± SD.

**Table 3:** Comparison of the QoR-9 scores (*x* ± *s*) of patients in the two groups.

	Group C	Group S	*p* value
*D*0	11.38 ± 2.47	13.05 ± 1.80	0.001^∗∗^
*D*1	15.10 ± 1.61	16.75 ± 1.50	0.000^*∗∗*^

^*∗∗∗*^=*P* < 0.01. Data are expressed as the mean ± SD.

**Table 4:** Incidence of severe cough (grades 2 and 3).

	Group C	Group S	*p* value
Just before extubation(bucking)	19 (47.5%)	9 (22.5%)	0.016^*∗*^

Postextubation			
10 min	11 (27.5%)	5 (12.5%)	0.028^*∗*^
1 h	5 (12.5%)	1 (2.5%)	0.054^*∗*^
4 h	0 (0%)	0 (0%)	0.062

^*∗*^=*P* < 0.05. Data are expressed as the number (% of total).

**Table 5:** Incidence of severe postoperative sore throat (POST) (grades 2 and 3).

	Group C	Group S	*p* value
30 min	23 (57.5%)	6 (15%)	≤0.001^∗∗^
2 h	14 (35%)	1 (2.5%)	≤0.001^∗∗^
4 h	7 (17.5%)	0 (0%)	≤0.001^∗∗^
24 h	2 (5%)	0 (0%)	≤0.001^∗∗^

^*∗∗*^=*P* < 0.01. Data are expressed as number (% of total).

**Table 6:** Incidence and severity of postoperative hoarseness of voice.

	Group C		Group S		*p* value
	Grade 2	Grade 3	Grade 2	Grade 3	
30 min	24 (60%)	16 (40%)	15 (37.5%)	25 (62.5%)	0.024^*∗*^
2 h	22 (55%)	13 (32.5%)	20 (50%)	16 (40%)	0.041^*∗*^
4 h	17 (42.5%)	11 (27.5%)	17 (42.5%)	10 (25%)	0.021^*∗*^
24 h	11 (27.5%)	7 (17.5%)	15 (37.5%)	2 (5%)	≤0.001^∗∗^

^*∗*^=*P* < 0.05; ^*∗∗*^=*P* < 0.01. Data are expressed as number (% of total).

**Table 7:** MAP comparison of two groups at different time points.

	Group C	Group S	*p* value
T0	98.58 ± 14.63	98.13 ± 12.45	0.883
*T*1	98.73 ± 16.39	88.93 ± 17.98	0.013^*∗*^
*T*2	94.43 ± 18.89	85.28 ± 14.54	0.017^*∗*^
*T*3	101.03 ± 14.99	87.75 ± 12.32	≤0.001^*∗∗*^
*T*4	92.80 ± 13.23	84.70 ± 11.31	0.004^*∗∗*^

^*∗*^=*P* < 0.05; ^*∗∗*^=*P* < 0.01. Data are expressed as mean ± SD.

**Table 8:** HR comparison of two groups at different time points.

	Group C	Group S	*p* value
*T*0	76.45 ± 13.46	75.35 ± 12.73	0.708
*T*1	84.75 ± 17.04	74.28 ± 13.54	0.003^∗∗^
*T*2	71.15 ± 12.69	67.78 ± 10.48	0.042^*∗*^
*T*3	80.48 ± 17.12	72.53 ± 12.42	0.020^*∗*^
*T*4	75.53 ± 13.80	70.20 ± 9.66	0.049^*∗*^

^*∗*^=*P* < 0.05; ^*∗∗*^=*P* < 0.01. Data are expressed as the mean ± SD.

## Data Availability

All data and materials are available without restriction. Researchers can obtain data by contacting the corresponding authors.
